# The therapeutic efficacy of I^131^-PSCA-mAb in orthotopic mouse models of prostate cancer

**DOI:** 10.1186/2047-783X-18-56

**Published:** 2013-12-13

**Authors:** Shengqiang Yu, Fan Feng, Ke Wang, Changping Men, Chunhua Lin, Qingzuo Liu, Diandong Yang, Zhenli Gao

**Affiliations:** 1 Department of Urology, Yantai Yuhuangding Hospital Affiliated to Medical College of Qingdao University, NO.20 East Yuhuangding Road, 264000 Yantai, China

**Keywords:** Radioimmunotherapy, Prostate cancer, Prostate stem cell antigen, Monoclonal antibody, Cell apoptosis

## Abstract

**Background:**

Prostate stem cell antigen (PSCA) is upregulated in prostate cancer tissues. Here we aimed to study the therapeutic efficacy of a monoclonal antibody of PSCA-labeled I^131^ (I^131^-PSCA-mAb) in orthotopic mouse models of prostate cancer.

**Methods:**

The proliferation, apoptosis and invasion abilities of PC-3 and LNCaP cells treated with I^131^-PSCA-mAb were measured by methyl thiazolyl tetrazolium assay, flow cytometry and transwell culture, respectively. The human prostate cancer models were established by orthotopic implantation of PC-3 and LNCaP cells in nude mice. I^131^-PSCA-mAb distribution and tumor cell apoptosis in the tumor-bearing nude mice were measured.

**Results:**

The inhibitory and apoptosis rates of PC-3 and LNCaP cells treated with I^131^-PSCA-mAb reached a maximum of 84%, 80% and 50%, 46%, respectively, which were obviously higher than in the cells treated with I^131^-IgG or PSCA-mAb. The invaded number of PC-3 and LNCaP cells treated with I^131^-PSCA-mAbe was significantly reduced (*P* < 0.01) compared with the control group. The ratios of I^131^-PSCA-mAb in tumor to intramuscular I^131^-PSCA-mAb (T/NT) in tumor-bearing nude mice were increased with time and reached the highest level after 8 h. T/NT stayed above 3.0 after 12 h, and the tumor could still be developed after 24 h. The number of apoptotic cells in tumor tissue of nude mice treated with I^131^-PSCA-mAb was larger than that in the control group.

**Conclusion:**

I^131^-PSCA-mAb has the potential to become a new targeted therapy drug for the treatment of prostate cancer.

## Background

Prostate cancer is one of the most frequently diagnosed malignancies worldwide and has become one of the leading causes of cancer-related death in men, only behind lung cancer [1,2]. Some patients with metastatic disease die within 2–3 years of diagnosis, whereas others with organ-confined disease can live for 10–20 years, which indicates that prostate tumors might have tremendous genomic diversity [3].

Androgens could contribute to the initial growth of prostate cancer [4]. In 1941, Huggins and Hodges successfully applied androgen deprivation therapy (ADT) by the injection of estrogens in metastatic prostate cancer patients in the form of surgical castration [5,6]. Within 1–2 years after initial response, progression of prostate cancer typically occurs; ADT could be considered as the treatment of choice for patients with advanced metastatic prostate cancer [7,8]. However, most prostate tumors ultimately progress to hormone-resistant prostate cancer (HRPC), which is androgen-independent growth, and resistance inevitably occurs within a few years, while antiandrogen therapy is initially effective [9]. Though early detection and treatment have improved significantly, biochemical recurrence might happen to almost 40% of men after radical retropubic prostatectomy [10]. The clinical manifestations of HRPC include increased concentrations of prostate serum antigen (PSA), bone metastases, soft-tissue/lymph node metastases and substantive pain [11].

Prostate stem cell antigen (PSCA) belongs to the Thy-1/Ly-6 family of the glycosylphosphatidylinositol-anchored cell membrane glycoprotein, which can overexpress in prostate cancer tissues [12]. Although PSCA expression has been detected in all stages of prostate cancer, the increased expression level of PSCA is positively correlated with biochemical recurrence, advanced stage, transition to the castration-resistant state and metastatic progression [13-16]. Ahmad et al. reported that a plasmid-based vaccine against PSCA may have the potential to be used in multimodal treatment programs for prostate cancer [17]. Saffran et al. found that administration of anti-PSCA mAbs could inhibit metastasis to distant sites and restrain the growth of established orthotopic tumor, which could significantly prolong the survival time of tumor-bearing mice [18]. However, the therapeutic outcomes using anti-PSCA mAbs for prostate cancer patients are very poor and limited. There are few studies on radioimmunotherapy guided by anti-PSCA mAbs for prostate cancer. The interesting area indicating the region of interest has been used in many surveillance systems, such as medical image processing [19].

In this study, anti-PSCA mAbs labeled with I^131^ (I^131^-PSCA-mAb) were made to investigate the potential therapeutic efficacy of I^131^-PSCA-mAb for prostate cancer. The proliferation abilities, apoptosis and invasion abilities of PC-3 and LNCaP cells treated with I^131^-PSCA-mAb *in vitro* were measured by methyl thiazolyl tetrazolium (MTT) assay, flow cytometry and transwell culture, respectively. Furthermore, human prostate cancer xenograft nude mice models were established by injection of androgen-dependent LNCaP cells and androgen-independent PC-3 cells. The distribution and variation of I^131^-PSCA-mAb in the tumor-bearing nude mice over time were measured by single-photon emission computerized tomography (SPECT) and the ROI method. Tumor cell apoptosis was detected by the terminal-deoxynucleotidyl transferase-mediated nick end labeling (TUNEL) technique.

## Methods

### Cell culture

Human prostate cancer PC-3 cell and LNCaP cell strains were purchased from Nanjing Keygen Biotechnology Co., Ltd. The PC-3 cells and LNCaP cells were maintained in RPMI-1640 and DMEM/F12 (GIBCO, USA) supplemented with 10% fetal calf serum (GIBCO, USA), respectively. All cells were incubated in a humidified air incubator with 5% CO_2_ at 37°C. The PC-3 cells and LNCaP cells at exponential growth phase were digested with 0.25% trypsin for inoculation.

### Animals

All animal studies were approved by the China Ethics Committee and performed in accordance with the ethical standards. A total of 15 12-week-old male nude mice (BALB/c-nu/nu) were recruited for the study. The male nude mice were from the Model Animal Research Center of Nangjing University. The nude mice were raised under the sterile barrier system with constant temperature (25-27°C) and humidity (40-50%) as well as experimental conditions accorded with the specific pathogen-free (SPF) standard. The nude mice were freely fed with high-pressure-sterilized forage and water.

### Establishment of prostate cancer models

The models of human prostate cancer were established in nude mice by orthotopic implantation. The PC-3 cells or LNCaP cells were inoculated into the anterior prostate of each nude mouse at the density of 2 × 10^7^ cells/ml. The 15 male nude mice were randomly divided into three groups: the group inoculated with 100 μl LNCaP cells (*n* = 5), the group inoculated with 100 μl PC-3 cells (*n* = 5) and the control group inoculated with 100 μl normal saline (*n* = 5).

### Labeling and identification of I^131^

The mouse anti-human PSCA IgG monoclonal antibodies (PSCA-mAb), which were specific to human orthotopic tumors in the mice and did not affect endogenous PSCA expression in these animals, were purchased from Sigma Co. in the USA. The labeling and identification of I^131^ in PSCA-mAb and control IgG were conducted at Shandong University.

### Measurements of cell inhibitory rate, apoptosis and invasion

The PC-3 and LNCaP cells were divided into four groups treated with normal saline, I^131^-PSCA-mAb, I^131^-IgG or PSCA-mAb, respectively. The difference in proliferation ability of PC-3 and LNCaP cells treated with the above three drugs including I^131^-PSCA-mAb, I^131^-IgG and PSCA-mAb (2 ug/ul) *in vitro* was measured by MTT assay. Briefly, 100 μl cells with the density of 2 × 10^4^ cells/ml was seeded into each well of a 96-well plate and incubated for 48 h. MTT (50 μl, 1 mg/ml) was added to each well, and the cells were incubated for 4 h. DMSO (150 μl) was later added to each well to solubilize the formazan crystals. The absorbance was read at 570 nm using a microplate reader. All determinations were carried out in triplicate. The inhibitory rate (IR) of the cell proliferation was calculated according to the equation: IR (%) = (1-A/A’) × 100% where A refers to the absorbance of the drug-treated group and A’ refers to the absorbance of the control group.

The difference in apoptosis of PC-3 and LNCaP cells treated with drugs *in vitro* was measured by an apoptosis assay kit according to the manufacturer’s instructions. AnnexinV-FITC (5 ul) was added to the cell suspension, and then propidium iodide (5 ul) was added after blending. The cells were incubated for 5–15 min at room temperature out of direct sunlight. Cell apoptosis was detected using flow cytometry (GUAVA, Millipore) within 1 h.

Cell invasion ability was determined using a transwell chamber (Corning, Mexico) with a pore size of 8.0 μm. Cells with the density of 1 × 10^5^ cells/ml in serum-free medium were added to each insert. After being cultured for 10 h at 37°C, the cells that had invaded the membrane were fixed by 4% paraformaldehyde and stained with 0.1% crystal violet. Five fields were selected randomly from the central and surrounding membrane, and then cells in every field were counted. All determinations were carried out in triplicate.

### SPECT for tumor-bearing nude mice

SPECT was performed on five tumor-bearing nude mice inoculated with androgen-independent PC-3 cells and five tumor-bearing nude mice inoculated with androgen-dependent LNCaP cells at 1 h, 4 h, 8 h, 12 h and 24 h after intravenous injection of 200 ul I^131^-PSCA-mAb (1 ug/ul) using a pinhole collimator. In order to block the uptake of I^131^ by the thyroid gland, nude mice were treated with a saturated solution of potassium iodide before the intravenous injection. The matrix was 128 × 128, and the zoom value was 1.33. The image data per frame were 2 × 10^5^ pixels. The ratio of I^131^-PSCA-mAb in tumor to intramuscular I^131^-PSCA-mAb (T/NT) in the tumor-bearing nude mice with time was measured using the ROI method with GE Xeleris software.

### Detection of tumor cell apoptosis

Apoptotic cells were detected by the TUNEL technique with an *in situ* cell death detection kit (Beyotime, China). The paraffin-embedded prostate tissues of the control group and experimental group were cut into 3-μm-thick sections and underwent routine deparaffinization and rehydration. Sections were incubated with the TUNEL reaction mixture containing terminal-deoxynucleotidyl transferase and label solution at 37°C for 1 h. Converted peroxidase (POD) was added later. 3, 3′-Diaminobenzidine (DAB) was used as a chromogen for final visualization.

### Statistical analysis

The measurement data were expressed as mean ± standard deviation and analyzed by *t*-test using SPSS version 17.0 software (Chicago, IL, USA). Differences were significantly statistical at *P* <0.05.

## Results

### Cell inhibitory rate

The inhibitory rates of PC-3 and LNCaP cells treated with drugs were measured by MTT assay (Figure 1). Compared with the control group, the proliferations of PC-3 and LNCaP cells treated with I^131^-PSCA-mAb, PSCA-mAb or I^131^-IgG were inhibited to different degrees. The inhibitory rates of PC-3 and LNCaP cells reached the maximum of 84% and 80%, respectively, when cells were treated with I^131^-PSCA-mAb. The inhibitory rates of PC-3 and LNCaP cells treated with I^131^-PSCA-mAb were significantly higher than those of the cells treated with PSCA-mAb or I^131^-IgG (*P* < 0.05).

**Figure 1:** **The inhibitory rates of PC-3 and LNCaP cells treated with I**^**131**^**-PSCA-mAb, I**^**131**^-IgG or PSCA-mAb (*P **< 0.05, compared with the LNCaP cells treated with I**^**131**^**-PSCA-mAb; #*P*** **< 0.05, compared with the PC-3 cells treated with I**^**131**^**-PSCA-mAb).**

### Cell apoptosis

The apoptosis of PC-3 and LNCaP cells treated with drugs *in vitro* was measured by flow cytometry (Figure 2). Compared with the control group, the apoptosis rates of PC-3 and LNCaP cells treated with I^131^-PSCA-mAb, PSCA-mAb or I^131^-IgG were gradually increased. The apoptosis rates of PC-3 and LNCaP cells reached the maximum of 50% and 46%, respectively, when cells were treated with I^131^-PSCA-mAb.

**Figure 2:** **The apoptosis of PC-3 and LNCaP cells treated with drugs.** (**a**: LNCaP cells treated with normal saline; **b**: LNCaP cells treated with PSCA-mAb; **c**: LNCaP cells treated with I^131^-IgG; **d**: LNCaP cells treated with I^131^-PSCA-mAb; **e**: PC-3 cells treated with normal saline; **f**: PC-3 cells treated with PSCA-mAb; **g**: PC-3 cells treated with I^131^-IgG; **h**: PC-3 cells treated with I^131^-PSCA-mAb).

### Cell invasion ability

The invasion ability of PC-3 and LNCaP cells treated with drugs was determined by transwell culture (Figure 3). Compared with the control group, there was no significant difference in the invasion ability between the group treated with PSCA-mAb and the group treated with I^131^-IgG. When cells were treated with I^131^-PSCA-mAb, the number of PC-3 and LNCaP cells that had invaded the membrane was 36 and 34, respectively. The number of invaded PC-3 and LNCaP cells treated with I^131^-PSCA-mAb was significantly lower than that of the control group (*P* < 0.01).

**Figure 3:** **The invasion abilities of PC-3 and LNCaP cells treated with I**^**131**^**-PSCA-mAb, I**^**131**^-IgG or PSCA-mAb (**P **< 0.01, compared with the cells treated with normal saline).**

### SPECT for tumor-bearing nude mice

The tumor-bearing nude mice inoculated with androgen-independent PC-3 cells or androgen-dependent LNCaP cells were examined by SPECT at 1 h, 4 h, 8 h, 12 h and 24 h after intravenous injection of I^131^-PSCA-mAb (Figure 4). The tumor developed clearly 1 h after intravenous injection, and the kidney, stomach and intestine had higher enhancement. The tumor enhancement region gradually increased over time, while the abdomen, blood and muscle enhancement decreased.

**Figure 4:** **The SPECT for tumor-bearing nude mice at 1 h, 4 h, 8 h, 12 h and 24 h after intravenous injection of I**^**131**^**-PSCA-mAb.** (**a**: tumor-bearing nude mice inoculated with androgen-independent PC-3 cells; **b**: tumor-bearing nude mice inoculated with androgen-dependent LNCaP cells).

The variation of I^131^-PSCA-mAb in the tumor-bearing nude mice over time was measured using the ROI method (Figure 5). The variation of T/NT with time was in accordance with the distribution *in vivo*. The T/NT of androgen-independent and androgen-dependent tumor-bearing nude mice increased with time and was highest at 4.2 and 4.4 after 8 h. The T/NT stayed above 3.0 after 12 h, and the tumor could still be observed after 24 h.

**Figure 5:** **The ratio of I**^**131**^**-PSCA-mAb in tumor to intramuscular I**^**131**^**-PSCA-mAb (T/NT) in the tumor-bearing nude mice at 1 h, 4 h, 8 h, 12 h and 24 h after intravenous injection of I**^**131**^**-PSCA-mAb.**

### Tumor cell apoptosis

The prostate tissue sections of the control and the experimental groups were analyzed by the TUNEL method to detect tumor cell apoptosis. There were apoptotic cells in androgen-independent and -dependent nude mice treated with I^131^-PSCA-mAb, and the number of TUNEL-positive cells was obviously larger than that in the control group (Figure 6).

**Figure 6:** **The tumor cell apoptosis of tumor-bearing nude mice treated with I**^**131**^**-PSCA-mAb.** (**a**: control group of androgen-dependent nude mice; **b**: androgen-dependent nude mice treated with I^131^-PSCA-mAb; **c**: control group of androgen-independent nude mice; **d**: androgen-independent nude mice treated with I^131^-PSCA-mAb).

## Discussion

PSCA is an ideal candidate for the detection or immunotherapy of prostate cancer because it has increased expression specificity for prostate cancer and has a specific cell surface location [12,20,21]. Radioimmunotherapy (RIT) uses monoclonal antibodies against tumor-specific antigens in conjunction with a particle-emitting radioisotope to deliver cytocidal ionizing radiation directly to the tumor [22]. In our study, the potential therapeutic efficacy of anti-PSCA mAbs in conjunction with I^131^ for prostate cancer was evaluated. We found that I^131^-PSCA-mAb showed great advantages in radioimmunotherapy and stronger positive anti-prostate tumor activity compared with I^131^-IgG and PSCA-mAb. Therefore, I^131^-based elimination of PSCA-producing cells seems to be a more efficient therapeutic method.

The immunotherapeutic efficacy of PSCA-mAb has been investigated by many studies considering PSCA as a putative target in a prostate cancer model, and the results of these studies have indicated that anti-PSCA antibodies have potential therapeutic roles for the treatment of prostate cancer [21,23]. In our study, we found that PSCA-mAb could inhibit the growth, apoptosis and migration of PC-3 and LNCaP cells to some extent. Therefore, these results are consistent with previous reports on anti-PSCA-based immunotherapy. RIT, which can target the corresponding antigens via binding radionuclides to antibodies, has a promising role in the treatment of metastatic melanoma, ovarian cancer and metastatic colorectal cancer [24-26]. The characteristic and complex interactions among the tumor, host, antigen-antibody complex and radionuclide determine the effectiveness of RIT [27]. In this study, the inhibitory and apoptosis rates of PC-3 and LNCaP cells treated with I^131^-PSCA-mAb reached up to the maximum of 84%, 80% and 50%, 46%, respectively, which were obviously higher than in the cells treated with I^131^-IgG or PSCA-mAb. Therefore, I^131^-PSCA-mAb could effectively inhibit the proliferation of cancer cells and promote the apoptosis of cancer cells. Compared with the control group, the number of invaded PC-3 and LNCaP cells treated with I^131^-PSCA-mAb was significantly reduced, which indicated that the invasion abilities of tumor cells were significantly reduced by I^131^-PSCA-mAb.

Furthermore, the ratios of I^131^-PSCA-mAb in tumor to intramuscular I^131^-PSCA-mAb (T/NT) in androgen-independent and -dependent tumor-bearing nude mice increased with time, which demonstrated that I^131^-PSCA-mAb-targeted radioimmunotherapy may have few or minimal undesired toxic effects on the other tissues. The T/NT stayed above 3.0 after 12 h, and the tumor could still be observed after 24 h. Therefore, guided treatment for prostate cancer could be precisely conducted. What is more, the number of apoptotic cells in androgen-independent or -dependent nude mice treated with I^131^-PSCA-mAb was larger than that in the control group. That is to say, I^131^-PSCA-mAb-targeted radioimmunotherapy could effectively promote cancer cell apoptosis in tumor-bearing nude mice. However, PSCA-mAb might not be able to specifically target non-PSCA-expressing tumor cells. Therefore, the applicability of I^131^-PSCA-mAb treatment in humans needs to be further explored.

## Conclusion

In conclusion, I^131^-PSCA-mAb has the potential to become a new targeted therapy drug for the radioimmunotherapeutic treatment of prostate cancer because it exhibited good targeting ability and efficacy and few side effects in nude mice models of human prostate cancer. We optimistically anticipate that I^131^-PSCA-mAb can be applied in clinical therapy.

## Competing interests

The authors declare that they have no competing interests.

## Authors’ contributions

SQY, DDY and ZLG designed the experiments. FF, KW and QZL carried out and interpreted the experiments. SQY, CPM and CHL wrote the article. All authors read and approved the final manuscript.

## Authors’ information

Shengqiang Yu and Fan Feng, the first two authors, should be regarded as joint first authors.
